The article "Deep Neural Networks for Optimal Selection of Features Related to Flu" was retracted in 2023. Reasons: signs of a paper mill; suspected computer-generated content; unreliable results or conclusions; concerns about the data.

# Deep Neural Networks for Optimal Selection of Features Related to Flu

**DOI:** 10.1155/2022/7639875

**Published:** 2022-07-14

**Authors:** B. Tarakeswara Rao, V. N. Lakshmana Kumar, D. Padmapriya, Kumud Pant, Tejaswini B, Wadi B. Alonazi, Khalid M. A. Almutairi, D.Raj, Ramesh Shahabadkar

**Affiliations:** ^1^Department of Computer Science & Engineering, Kallam Haranadhareddy Institute of Technology, Dasaripalem, Andhra Pradesh 522019, India; ^2^Department of Electronics and Communication Engineering, M.V.G.R.College of Engineering (Autonomous), Vizianagaram, Andhra Pradesh 535005, India; ^3^Department of Electronics and Communication Engineering, Panimalar Engineering College, Chennai, Tamil Nadu 600123, India; ^4^Department of Biotechnology, Graphic Era Deemed to Be University, Dehradun, Uttarakhand 248002, India; ^5^Department of Information Science and Engineering, East Point College of Engineering and Technology, Bengaluru, Karnataka 560049, India; ^6^Health Administration Department, College of Business Administration, King Saud University, P.O. Box. 71115, Riyadh 11587, Saudi Arabia; ^7^Department of Community Health Sciences, College of Applied Medical Sciences, King Saud University, P.O. Box. 10219, Riyadh 11433, Saudi Arabia; ^8^Zoonosis Research Center, School of Medicine, Wonkwang University, Iksan, Republic of Korea; ^9^Department of Electrical and Computer Engineering, Ambo University, Woliso Campus, Waliso, Ethiopia

## Abstract

In recent times, humans who have been exposed to influenza A viruses (IAV) may not become hostile. Despite the fact that KLRD1 has been discovered as an influenza susceptibility biomarker, it remains to be seen if pre-exposure host gene expression can predict flu symptoms. In this paper, we enable the examination of flu using deep neural networks from input human gene expression datasets with various subtype viruses. This study enables the utilization of these datasets to forecast the spread of flu and can provide the necessary steps to eradicate the flu. The simulation is conducted to test the efficiency of the model in predicting the spread against various input datasets. The results of the simulation show that the proposed method offers a better prediction ability of 2.98% more than other existing methods in finding the spread of flu.

## 1. Introduction

Coronavirus 2019, which is highly contagious and severe, is considered a common respiratory illness after influenza (flu). Infections with the influenza A virus (IAV) account for approximately 75% of infections [1–4]. Adults have been infected with the IAV at a rate of 2.3%. However, not everyone who is exposed to the virus becomes ill [5]. The majority of young people, slightly more than half, become infected with IAV and develop respiratory tract symptoms; the other half either does not develop symptoms or does not get infected at all when given a controlled IAV exposure [6–8]. The fact that influenza has such a substantial influence on the economy and peoples' health [9–11] makes it imperative to predict who will become ill and when. If IAV-infected people are not identified and treated promptly, the number of deaths will rise as a result of increased viral transmission and, possibly, worsening of sickness [12, 13]. On the other hand, influenza vaccines may not be effective for all people [14], despite the fact that immunisation is recommended for the prevention of the flu as well as the promotion of public health among hospitals, educational institutions, societies, and communities. An alternate method of controlling the spread of IAV and reducing mortality as a result of IAV and its sequelae would be to anticipate who would get infected before they are exposed to the virus.

The article "Deep Neural Networks for Optimal Selection of Features Related to Flu" was retracted in 2023. Reasons: signs of a paper mill; suspected computer-generated content; unreliable results or conclusions; concerns about the data.

It is not known whether gene expression in the host before exposure to IAV can predict susceptibility to the virus. When it comes to predicting influenza susceptibility, KLRD1 expression has recently been discovered to be the polar opposite of what was previously thought. In addition, two prediction models for predicting host sensitivity to RSV have yielded promising findings [15] in terms of anticipating host sensitivity to RSV. The major possibility is to use a support vector regression model [16] with an RBF kernel and learn directly from host gene expression. One of the methods uses biological routing that gets derived from the gene datasets [17] of the Signature database. The regularized regression LASSO method [18] similarly uses biological pathway modulation and is derived from the Molecular Signature Database (MSigDB). There has been no evidence to demonstrate that advanced machine learning algorithms can consistently forecast the IAV onset infections before the exposure of viral infections, or if they can outperform the KLRD1 biomarker in predicting the onset of infection.

The gene expression to identify IAV infection before its symptoms occur is distinct from the gene expression to forecast the host susceptibility to the virus. Several factors, including immune memory [19], genetics, circadian and seasonal shifts [20], gender [15], age [21], and time of day [22], all influence both host gene expression responses, though they do so at different times. Assuming that IAV susceptibility can be predicted by examining the period of time preceding an exposure, it may be able to identify the hosts that have been infected with the virus both before and after the exposure has occurred. The detection of IAV infection by measuring the host gene expression has proven to be a successful strategy. IAV infection can be detected using gene expression profiles in the peripheral blood that are distinct from those seen in viral, respiratory, and bacterial infections. With greater than 90% accuracy, these gene expression profiles were applied with real-time affected cases of the H1N1 pandemic.

The article "Deep Neural Networks for Optimal Selection of Features Related to Flu" was retracted in 2023. Reasons: signs of a paper mill; suspected computer-generated content; unreliable results or conclusions; concerns about the data.

While the data is compared with the top 50 genes using latent factor regression analysis from discriminative factors, it is possible to find cross-strain IAV infection signatures. This is because IAV substrain infection signatures are so similar. According to a multicohort study [15], out of the 50 genes, certain genes (11 genes) from influenza can be utilised to identify symptomatic patients infected with IAVs. In order to determine whether a similar level of effectiveness can be obtained in anticipating host sensitivity to IAV, it is necessary to answer the question. According to the findings of this research, deep neural networks can be utilised to investigate flu by using human gene expression datasets as input as well as a range of virus subtypes as training data. Using these numbers, the researchers hope to be able to anticipate flu epidemics and develop the tactics necessary to eradicate the disease. In order to determine the model's ability to forecast the spread, it is tested against a range of input datasets.

The main contribution of the paper involves the following:

- The authors enable the examination of flu using deep neural networks from the input human gene expression datasets with various subtype viruses
- The study enables the utilization of these datasets to forecast the spread of flu and can provide the necessary steps to eradicate the flu

The outline of the paper is given as follows: Section 2 discusses the related works; Section 3 provides the details of the proposed work; Section 4 evaluates the entire work; Section 5 concludes the work with possible directions of future scope.

## 2. Related Works

In order to accurately and effectively evaluate the associations between influenza-like sickness and air quality data, the study in [16] presented an air quality data analysis. They were able to establish a new integrated platform by merging Hadoop and Spark in a cluster environment. The relationship between influenza-like illness and poor air quality was also demonstrated and discussed. In a study conducted by the author [17], invasive aspergillosis was found to be associated with fine particle air pollution. According to the findings of this study, there is a relationship between PM2.5 concentration and aspergillosis occurrence.

The article "Deep Neural Networks for Optimal Selection of Features Related to Flu" was retracted in 2023. Reasons: signs of a paper mill; suspected computer-generated content; unreliable results or conclusions; concerns about the data.

The authors in [18] have shown the feasibility of RNN-based analysis and forecasting of air pollution. In this project, we used RHadoop to build a distributed computing system for analysing air pollution and displaying a visualisation of historical data using the HBase data storage. In this paper, a forecast for PM2.5 was presented on the basis of the MAPE, with its accuracy measured and discussed. [19] developed a data analysis in an integrated way to determine the relationship between the Air Quality Index (AQI), climatic conditions, and respiratory infection risk. As a consequence of their research, they discovered that a decrease in ILI cases is statistically linked to an increase in the Air Quality Index (AQI) that in turn lowered the risk of lung disease by up to three days.

Authors in [20] used LSTM-RNNs for the estimation of influenza trends, and the results were promising. These researchers used a range of new data sources to forecast influenza trends in the beginning, including viral monitoring, regional influenza propagation, , environmental and air pollution levels, and other data sources such as Google trending topics. Researchers discovered a strong relationship in terms of the incidence of ILI and a variety of environmental and climatic variables.

According to [21], influenza epidemics were forecasted using multistep LSTM prediction models. As a result, it was discovered that an LSTM framework was the most accurate when it came to creating single-output predictions. From stages 2 to 13, the MAPE for ILI rates in the United States of America was 12.930% on average. When compared to other machine learning models, it was discovered that the proposed CNN-LSTM has the highest projected accuracy, which was confirmed. The CNN-LSTM model was also put through its paces to investigate if it could accurately estimate the PM2.5 concentration. The authors in [22] suggested an LSTM-based technique for estimating PM2.5 concentrations, which makes use of RNNs to make their predictions. A neural network was constructed and RNNs employing LSTM were executed using Keras, where they collected training data for the network and transformed it into 20-dimensional data. A group of scientists conducted experiments with PM2.5 levels in order to determine how essential they were over the next four hours. The proposed technique was successful in predicting PM2.5 levels with high accuracy.

Using large amounts of environmental data and deep learning, they have developed new algorithms for calculating pollution concentrations. In order to incorporate enormous volumes of data, the approach makes use of two types of deep networks. The features of the input data are automatically extracted using a convolutional neural network, which serves as the design foundational layer. The time dependence of pollutants was determined by incorporating a long-term memory network onto the output layer. It was possible to anticipate future PM2.5 concentrations by using performance time-series optimization. In the end, it was discovered that the forecasts and the numerical model testing were related. In addition, the model utility and application were thoroughly investigated. As a result of the experiments, it was discovered to be more accurate than typical models.

The article "Deep Neural Networks for Optimal Selection of Features Related to Flu" was retracted in 2023. Reasons: signs of a paper mill; suspected computer-generated content; unreliable results or conclusions; concerns about the data.

## 3. Proposed Method

Here, the study goes through the RNN, LSTM, and mean absolute percentage error (MAPE). These are all components of our overall strategy in further detail. This section delves deeper into the specifics of each individual component in greater depth.

### 3.1. Recurrent Neural Network (RNN)

An RNN is considered a neural network, which is a network type that merely feeds the network output into the system rather than the other way around. As a result of this technique, the memory of the neural network is improved. The architecture of a RNN is illustrated in Figure 1. The RNN architecture involves the input to be acquired from its previous layer, and then, subsequently, the weights are assigned to estimate the flu from the input feature extraction instances.

The output of the web is retained between each round of processing and until the next transfer procedure is performed. The conclusion derives from this: whenever we talk about time, the study is actually talking about t+1 points. It is taken into consideration, and as a result, it has the characteristics of a memory that exists both before and after the input.

The RNN may be determined by using the following equation:

(1) $$\begin{array}{c} ht=\sigma h\left(Whxt+Uhyt-1+bn\right), \end{array}$$

(2) $$\begin{array}{c} yt=\sigma y\left(Wyht+by\right), \end{array}$$

where xt is the input layer vector, ht is the hidden layer vector, yt is the output layer vector, *W*, *U*, and *b* are the matrix or the vector of the weight parameter, and *σ*h and *σ*y are the activation functions.

As it can be seen from this formula, the output of the time unit before yt1 is included in the yt−1 calculation.

### 3.2. Long Short-Term Memory Network

Because of the addition gate mechanism, the LSTM is capable of successfully storing events that occur before the long-distance time, even when the RNN is used as the basis for the model. The weights of this technique are able to correct the gradient disappearance issue of the random neural network. This is why LSTM is more suited for processing significant time-series events that occur at more frequent intervals than the RNN (Figure 2).

The article "Deep Neural Networks for Optimal Selection of Features Related to Flu" was retracted in 2023. Reasons: signs of a paper mill; suspected computer-generated content; unreliable results or conclusions; concerns about the data.

As previously stated, the LSTM formula is as follows:

(3) $$\begin{array}{c} it=\sigma \left(Wiht-1+Uixt+bi\right), \end{array}$$

(4) $$\begin{array}{c} ft=\sigma \left(Wfht-1+Ufxt+bf\right), \end{array}$$

(5) $$\begin{array}{c} ot=\sigma \left(Woht-1+Uoxt+bo\right), \end{array}$$

(6) $$\begin{array}{c} ct=\tan h\left(Wht-1+Uxt+b\right), \end{array}$$

(7) $$\begin{array}{c} ct=ft\cdot ct-1+it\cdot ct, \end{array}$$

(8) $$\begin{array}{c} ht=ot\cdot \text{Tan}h\left(ct\right), \end{array}$$

(9) $$\begin{array}{c} yt=ht, \end{array}$$

where *h*_*t*_ is the gate to find if the input value is sent to the memory state, *f*_*t*_ is the gate to find if the forgot gate is previously sent and recorded at the memory state, and *o*_*t*_ is the output gate that influences the output of the memory to the hidden layer.

### 3.3. MAPE

The MAPE of a measurement can be used to determine the precision of the measurement. Another way of putting it is that the MAPE is expressed as a percentage, making it easier for the process of understanding the precision metrics. Despite the fact that the model appears to match the data precisely, a significantly high MAPE value may still be noticed. Examine the graph to see if there are any data points that are near the zero-point boundary. Because it is divided by the actual data over the absolute error, the MAPE causes the MAPE to be exaggerated by a significant amount.

## 4. Results and Discussions

For this project, the RNN made use of the following factors and methodologies: the activation function of a rectified linear unit (ReLU) is used in hidden and input layers because it proved to be capable of overcoming the vanishing gradient. The output layer translated it into a binary choice with a strictly rising [0, 1] outcome by employing a logistic regression in the input layer. Adam has the potential to perform well in parameter spaces. Cross-validation on the source dataset, as well as external validation, was utilised to evaluate the performance of the RNN.

Figures 3–7 illustrate the performance of predictive modelling algorithms that employ the entire 22,277 array probes and are divided randomly into training (80%) and testing (20%) data. The majority of the research included in this investigation used training and testing data that was not restricted to the data collected prior to exposure. Using all three models, including RNN, RF, and SVM, it is possible to learn the specific gene expression signals of the influenza virus. As a result, RNN will serve as the foundation for all future RNN developments.

The article "Deep Neural Networks for Optimal Selection of Features Related to Flu" was retracted in 2023. Reasons: signs of a paper mill; suspected computer-generated content; unreliable results or conclusions; concerns about the data.

Cross-validation is used to compare RNNs that have been trained over a variety of time periods starting at the beginning (the day before exposure) and progressing until the point of exposure as shown in Figures 3–7. Another way of putting it is that the only data stored in T0 is the expression data, which has not been exposed to a virus yet.

It was discovered that when only 4,164 of the 22,277 features were employed, the RNN performance was inferior to that achieved when all 22,277 features were used. Its overall performance was not diminished as a result of this. Specifically, all four models that used the most important IAV postinfection discriminative genes failed miserably. There were no good AUROC or AUPR values for the four H1N1 models that used a limited gene set because the gene set used was too small. Regarding H3N2, the models were just modestly more accurate than a blind estimate in this particular instance.

Diagnosing overfitting in the RNN was accomplished using cross-validation. Each RNN model was built in the same way, with the exception of the hidden layer nodes, which varied from model to model. While the model may have performed well on the training set, we looked for instances where the model failed to predict new occurrences when evaluated on a different dataset.

Deep learning has been proven to be capable of predicting whether a person would contract the flu quickly after being exposed to IAV before the exposure, as demonstrated by cross-validation and external validation data in this study. This study's findings are consistent with previous research [7, 15]. According to the findings of all of the studies, it is feasible to anticipate a person's sensitivity to viral respiratory diseases. The reduction of dropout rates enables the models to achieve a wide range of classified instances from the feature selected instances, where the rate of classification errors has reduced to the core than the other existing methods.

We demonstrate that deep learning can be used to analyse gene expression data even when the data is not of the typical large size. In order to forecast influenza susceptibility without overfitting, it was discovered that an RNN with 100 hidden layers and 100 nodes per layer was the most effective as in Figure 4. In order to avoid overfitting RNN on holdout data, dropout is used as a regularisation step, and cross-validation is used to select the most robust model.

When it comes to predicting IAV vulnerability, selecting the appropriate features can be critical. Among the biomarkers, only the KLRD1 biomarker outperforms the RNN. However, our findings suggest that larger feature sizes result in an improved prediction performance in general. The optimum model is to make use of all 22,274 RNN features available. Considering that the RNN model exploited the hallmark genes of MSigDB, which accounted for only one-fifth of the total features, it is possible that only a small number of candidate genes directly connected to an individual sensitivity to IAV exist within it. However, it is possible that a more intricate molecular mechanism may be necessary to properly comprehend the selected features. However, as a result, the complete set of characteristics proved to be a superior substitute. There were insufficient genes to fix this problem. Only a small number of IAV infection genes were used in the models, and these models consistently underperformed the others.

The article "Deep Neural Networks for Optimal Selection of Features Related to Flu" was retracted in 2023. Reasons: signs of a paper mill; suspected computer-generated content; unreliable results or conclusions; concerns about the data.

The data also demonstrates that the RNN model beats the other three models in terms of recognising patterns of gene expression associated with immunity for IAV, according to the researchers. The reason why expecting H3N2 susceptibility is superior to forecasting H1N1 susceptibility is still up in the air, and no definitive answer has been provided. When it comes to H3N2 and H1N1, the peak of symptoms occurs after infection. Therefore, we assume that the length of the latency phase is a factor [7].

Perhaps T0 gets closer with H3N2 symptoms than its H1N1 onset; the H3N2 models are more accurate than the H1N1 models. A further factor that may be important is the difference in the proportions of H3N2- and H1N1-infected people. 32% of the validation data indicates that this is not the case. An increase in the number of infected patients could have a negative impact on the performance of the H1N1 virus model.

It is also critical to understand when you should train. According to the findings of this study (T0), the best results appear to have been obtained when data were collected during the same time period prior to exposure. A consequence of this is that if different time periods are employed, the performance may degrade.

## 5. Conclusions

According to the findings of this research, deep neural networks can be utilised to investigate flu by using human gene expression datasets as input as well as a range of virus subtypes as training data. Using these numbers, the researchers hope to be able to anticipate flu epidemics and develop the tactics necessary to eradicate the disease. In order to determine the model's ability to forecast the spread, it is tested against a range of input datasets. Through the use of a computer simulation, we were able to demonstrate that our technique is more accurate in predicting flu epidemics than the alternatives. There may yet be room for improvement in the field of prediction. It is possible that increasing the amount of training data available by mixing the H1N1 and H3N2 records will not result in better prediction results in the long run. Based on the RNN performance when using mixed data, it is possible that there are distinct distinctions between influenza A (IAV) strains in terms of susceptibility to the virus.

The article "Deep Neural Networks for Optimal Selection of Features Related to Flu" was retracted in 2023. Reasons: signs of a paper mill; suspected computer-generated content; unreliable results or conclusions; concerns about the data.

There are some flaws in this study that need to be addressed. To begin with, little research has been conducted to investigate the gene expression patterns of influenza virus strains. If you have a large amount of gene expression data, you may be able to improve the performance of your RNN even more. A second aspect to mention is that it is unclear whether the subjects had already been infected with IAV. It may be required to make changes to these variables in order to conduct a more accurate comparison or validation of results. Finally, the molecular mechanisms that underlie IAV vulnerability or immunity are still not fully known, as previously mentioned. In the future, various other models can be used for finding the immunity and vulnerability associated with gene expression datasets collected from various repositories.

## Figures and Tables

**Figure 1:** RNN architecture.

**Figure 2:** LSTM schematic diagram.

**Figure 3:** Accuracy.

**Figure 4:** Sensitivity.

**Figure 5:** Specificity.

**Figure 6:** Precision.

**Figure 7:** AUROC.

## Data Availability

The data used to support the findings of this study are included within the article. Further data or information is available from the corresponding author upon request.
